The article "Ultrasound Images Guided under Deep Learning in the Anesthesia Effect of the Regional Nerve Block on Scapular Fracture Surgery" was published in 2021. Journal: J Healthc Eng.

# Ultrasound Images Guided under Deep Learning in the Anesthesia Effect of the Regional Nerve Block on Scapular Fracture Surgery

**DOI:** 10.1155/2021/6231116

**Published:** 2021-10-07

**Authors:** Yubo Liu, Liangzhen Cheng

**Affiliations:** ^1^Department of Anesthesiology, Jiangxi Armed Police Corps Hospital, Nanchang 330000, Jiangxi, China; ^2^Second Department of Surgery, Jiangxi Armed Police Corps Hospital, Nanchang 330000, Jiangxi, China

## Abstract

In order to discuss the clinical characteristics of patients with scapular fracture, deep learning model was adopted in ultrasound images of patients to locate the anesthesia point of patients during scapular fracture surgery treated with the regional nerve block. 100 patients with scapular fracture who were hospitalized for emergency treatment in the hospital were recruited. Patients in the algorithm group used ultrasound-guided regional nerve block puncture, and patients in the control group used traditional body surface anatomy for anesthesia positioning. The ultrasound images of the scapula of the contrast group were used for the identification of the deep learning model and analysis of anesthesia acupuncture sites. The ultrasound images of the scapula anatomy of the patients in the contrast group were extracted, and the convolutional neural network model was employed for training and test. Moreover, the model performance was evaluated. It was found that the adoption of deep learning greatly improved the accuracy of the image. It took an average of 7.5 ± 2.07 minutes from the time the puncture needle touched the skin to the completion of the injection in the algorithm group (treated with artificial intelligence ultrasound positioning). The operation time of the control group (anatomical positioning) averaged 10.2 ± 2.62 min. Moreover, there was a significant difference between the two groups (*p* < 0.05). The method adopted in the contrast group had high positioning accuracy and good anesthesia effect, and the patients had reduced postoperative complications of patients (all *P* < 0.005). The deep learning model can effectively improve the accuracy of ultrasound images and measure and assist the treatment of future clinical cases of scapular fractures. While improving medical efficiency, it can also accurately identify patient fractures, which has great adoption potential in improving the effect of surgical anesthesia.

## 1. Introduction

Scapular fracture was first described by Desault in 1805, who studied the characteristics of scapular fracture. Scapular fracture accounts for 1% of total body fractures and 5% of total shoulder fractures [1]. It is usually caused by accidents such as car accidents or falling from heights. The majority of young men and middle-aged men account for 64% to 90% [2]. Scapular fractures such as painful fractures and fall fractures (fatigue injuries) are rare. Scapular fracture is often part of multiple traumas and is often overlooked. With the development of society, science and technology, and transportation, its incidence is gradually increasing [3]. A combination of physical examination, x-ray, or CT examination can usually make a definitive diagnosis of shoulder and foot fractures. At present, most of the surgical treatments for scapular fractures focus on the shoulders, kidneys, and neck, including the articular surfaces, which need to be reduced anatomically as much as possible. However, the incidence of postoperative complications such as joint pain, instability, and shock is relatively high [4].

The local nerve block is mainly used for surgical anesthesia of the shoulder and wrist area. The requirements of local nerve block for patient's systemic physiological functions and hardware equipment are lower compared with general anesthesia, and postoperative pain relief is relatively less [5]. In addition, the local nerve block can reduce general anesthesia. In areas where the local nerve distribution is relatively concentrated, the local nerve block mainly forms various block paths, including muscle groove, subclavian, subclavian longitudinal penetration, subclavian polymorphic process, and axillary path [6]. The operation of traditional nerve fracture surgery requires that the patient should be awake and can assist to report feelings, and the puncture needle of the nerve trunk is contacted within a short period of time, which will cause the patient's subjective discomfort and may cause nerve damage during the puncture process [7]. The key to the success of nerve fracture surgery is the correctness of the position of the peripheral nerve. It requires the surgeon's high clinical experience, which has a great impact on the patient's various anatomical changes, so the success rate is not high. Nerve fracture surgery is often accompanied by lesions of blood vessels or important tissues and organs, which may cause serious complications or sequelae. The development and application of nerve stimulation devices have increased the success rate of nerve fracture surgery. However, puncture increases the discomfort of patients, and the use of intravenous analgesics and sedatives is gradually increasing [8]. In recent years, with the advancement of medical technology and the improvement of human medical treatment, the demand for rapid onset, long-term maintenance, high success rate, and uncomplicated nerve fracture surgery has also increased. With the help of the anatomical positioning of the nerve stimulator, the peripheral nerve block becomes wider and wider. In recent decades, the emergence of ultrasonic technology has made scapular fracture surgery safer and more effective and further expanded the scope of application [9]. This technology rapidly changed the way of clinical anesthesia, and local anesthesia can be performed in a visualized manner. Ultrasound is dynamic, real-time, recordable, and radiation-free, and ultrasound-guided nerve block technology has been developing and maturing in the past decade [10]. Ultrasound-guided nerve block is different from conventional techniques. Traditional methods identify target nerves by looking for paresthesia methods through body surface anatomical location or inducing neuromuscular contraction by nerve stimulator, but traditional methods cannot achieve visualization of puncture points [11]. Ultrasound imaging can visualize the nerve that needs to be blocked, as well as the accompanying blood vessels and important tissues around the nerve. By visualizing the nerve and the important structures surrounding the nerve, it is possible to ensure accurate diffusion of anesthetic drugs around the target nerve during nerve block. It also avoids damage to blood vessels and surrounding important tissue structures and reduces the incidence of adverse events such as intrathecal injection and intravascular injection [12].

Deep learning is a new research direction in the field of machine learning. Unlike traditional machine learning, deep learning neural networks include many hidden layers. The machine can automatically learn the characteristics of each level of the data and completely analyze and process the data information. The excellent results of deep learning technology in the medical field are mainly reflected in the processing and analysis of medical images [13]. It does not need to manually extract the function or preprocess the image. It can extract the information in the image and the depth features of the image, thus contributing to disease diagnosis and diagnosis. At present, the research and application of in-depth learning in the field of anesthesia are relatively rare, and the risk of death of patients after general anesthesia can be predicted based on the data extracted during surgery. In addition, deep learning has broad application prospects for its performance and scalability in anesthesia research.

The purpose of this research was discussing the following three issues: first, the difference in image accuracy between deep learning ultrasound images and ordinary ultrasound images; second, the adoption of artificial intelligence ultrasound to optimize anesthesia puncture path; third, the effectiveness of ultrasonographic imaging guided scapular regional nerve block in the treatment of surgical pain of fracture. It was hoped to provide reference for other regional nerve block anesthesia operations.

## 2. Methods

### 2.1. Research Objects

In this study, a total of 100 patients with scapula surgery who underwent surgery from July 2017 to July 2019 were recruited. This study had been approved by the Medical Ethics Committee of the Hospital, and the family members of the patients included in the study had signed the informed consent form.

  Inclusion criteria were as follows: (i) patients with diseases such as hypertension, diabetes, and respiratory insufficiency according to the standards of the *American Society of Anesthesiology (ASA)*; (ii) scapular fracture surgery not exceeding four hours
  Exclusion criteria were as follows: (i) patients with paralysis; (ii) patients with speech dysfunction; (iii) patients with skin infection at the puncture site; (iv) patients with arm nerve plexus injury; (v) patients with previous clavicle surgery experience; (vi) patients with pleural fluid or ascites

In 100 patients undergoing scapular surgery, 1% of the local anesthetic concentration and 7% of Lopimaran were injected into the area to be anesthetized. Patients were randomly rolled into control group (traditional body surface positioning) and algorithm group (ultrasound-guided positioning).

### 2.2. Experimental Environment

#### 2.2.1. Construction of the Deep Learning Segmentation Model

Convolutional neural network is a commonly used deep learning algorithm [14]. The process is as follows. Triggered by the human visual system, the continuous modification is formed in a multilayer neural network suitable for processing and recognizing images. A classic convolutional neural network is composed of a convolutional neural layer and a normalization layer, and its structure is shown in Figure 1.

## 3. SegNet Model

Seg is a brand-new deep fully convolutional neural network model (semantic pixel-wise neural network model) proposed by three deep learning experts (Yadri-narayanan, Kcndall, and Cipolla) from the University of Cambridge in 2010 that can perform image pixel-wise semantic division and image labeling [15]. The SegNet model is mainly composed of encoder, decoder, and oft-max layer. The encoder and decoder appear in pairs for image feature extraction and optimization. Its structure is shown in Figure 2.

The SegNet model divides an image into low-frequency part, which is obtained by low-pass filtering (smoothing and blurring) of the image, and high-frequency part, which is obtained by subtracting the low-frequency part from the original image [16]. The goal of the algorithm is enhancing the high-frequency parts that represent details, that is, multiplying the high-frequency parts by a certain gain value and then recombining them to obtain an enhanced image. Therefore, the core of the SegNet model is the calculation of the high-frequency part of the gain coefficient. One solution is setting the gain to a fixed value, and the other solution is expressing the gain value as a quantity related to the variance, which will be explained in the additional equation later.

It is assumed that the pixels in an image are represented as *x*(*i*, *j*); then with (*i*, *j*) as the center, in the area where the window size is (2*n* + 1) ∗ (2*n* + 1), its local mean sum and variance can be expressed as the following equations:

(1) $$\begin{array}{c} m_{x}\left(i,j\right)=\frac{1}{{\left(2n+1\right)}^{2}}\sum_{k=i-n}^{i+n}\sum_{l=j-n}^{j+n}x\left(k,l\right),\\ \sigma_{X}^{2}\left(i,j\right)=\frac{1}{{\left(2n+1\right)}^{2}}\sum_{k=i-n}^{i+n}\sum_{i=j-n}^{j+n}{\left[x\left(k,l\right)-m_{x}\left(i,j\right)\right]}^{2}. \end{array}$$

The mean value *mx* can be approximately regarded as the background part, at this time *x-m* is the high-frequency detail part, and the gain product for the high frequency is the following equation:

(2) $$\begin{array}{c} f\left(i,j\right)=m_{x}\left(i,j\right)+G\left(i,j\right)\left[x\left(i,j\right)-m_{x}\left(i,j\right)\right]. \end{array}$$

For the gain *G*, the first option is taking a constant greater than 1 to achieve the enhanced effect, which is the following equation:

(3) $$\begin{array}{c} f\left(i,j\right)=m_{x}\left(i,j\right)+C\left[x\left(i,j\right)-m_{x}\left(i,j\right)\right]. \end{array}$$

Option two is that it is expressed as a change value inversely proportional to the local mean square error, which is the following equation:

(4) $$\begin{array}{c} f\left(i,j\right)=m_{x}\left(i,j\right)+\frac{D}{\sigma_{x}\left(i,j\right)}\left[x\left(i,j\right)-m_{x}\left(i,j\right)\right]. \end{array}$$

The local mean square error is large in the high-frequency area of the image, and the gain value is small at this time, so that the result will not be too bright. However, the local mean square error is very small in the smooth area of the image, and the gain value is large at this time, which may amplify the noise signal. Therefore, it is necessary to limit the maximum gain to get better results.

### 3.1. Adaptive Contrast Enhancement

The principle of this network is classifying the image into two parts. The low-frequency part can be obtained by low-pass filtering of the image. The high-frequency part is obtained by subtracting the low-frequency part from the original image. The purpose of this algorithm is visualizing the image in detail, that is, multiplying the high-frequency part by a certain gain value to reconstruct the emphasized image. The core of enhancing image accuracy is repeatedly enlarging clear images in order to improve image quality.

Nowadays, medically generated images are mainly concentrated on low-frequency components, while noise and image details are concentrated on high-frequency components. The two components are separated in image processing, and different operations and processing are performed, which can avoid image detail loss and noise amplification when the histogram equalization algorithm is used. It aims to separate the high-frequency and low-frequency components of the input image. Medical ultrasound images have detailed and strict requirements, and blurring is not allowed, so Gaussian low-frequency filters were used in this study.

### 3.2. Anesthesia Methods

4-5 *μ*g/kg fentanyl, 1.5–2 mg/kg propofol, and 0.1 mg/kg vecuronium were used. After successful tracheal intubation, the anesthesia machine was connected to mechanical ventilation, the tidal volume was 8–10 mL/kg, and the respiratory rate was 8–12 times/min. During the operation, 0.06–0.1 *μ*g/kg/min remifentanil was used for continuous intravenous pump injection, Sevoflurane 1.0–1.3 MAC inhalation maintained the depth of anesthesia within 40–60 BIS value, and intermittent intravenous injection of vecuronium was made to maintain muscle relaxation. If the heart rate was lower than 55 beats/min, 0.3 mg atropine was given, and when the systolic blood pressure was lower than 25% of the preoperative base value, 10 mg ephedrine was given to increase blood pressure.

### 3.3. Traditional Body Surface Localization of the Scapula Regional Nerve Block

The patient was anesthetized on the inner side and 1/3 of the unaffected side of the site to be anesthetized. The patient was supine with the head tilted to about 1.5–2.0 cm. After disinfection of the scapular fracture site, a 20 g puncture needle was inserted along the muscularly groove, and the needle was slowly inserted in the lower and lateral directions. The needle was inserted 1.5 to 2.0 cm, and the patient can feel the pain and location of the puncture, so that the physician was informed. 20 mL local anesthetic was injected into the muscle, and a 5-minute massage was made to spread the anesthetic fluid further away.

### 3.4. Artificial Intelligence Ultrasound-Guided Scapula Regional Nerve Block

The patient was anesthetized on the inner side and 1/3 of the unaffected side of the site to be anesthetized. The head should be tilted to about 1.5–2.0 cm and the patient should be supine with the scapula fracture in contact. After disinfection, ultrasound was used to detect the nerves that needed to be anesthetized. It was relatively more pronounced by detecting the neural structure at the margin lateral margin of the scapula. After the ultrasound showed the nerves at the anesthetic site, the location of the puncture should be determined and a local anesthetic of 20 mL was injected into the muscle. After 5 minutes of massage, the anesthetic fluid spread further.

### 3.5. Observation Indexes

The operative time, puncture depth, puncture adjustment time, time to start anesthesia, rate of good anesthesia, complication rate, and other indicators of the two localized nerve area approaches were shown. (I) The time of blocking action referred to the time from the contact with the skin of the puncture needle to the completion of the injection. The measuring tool of the ultrasonic device was used to measure the distance from the puncture point to the target, and the actual puncture depth was measured with a carrier. (II) The needle adjustment times during the puncture process were recorded, so did the occurrence of bone, needle head, and needle body defects during the puncture process. In addition, the number of cases of loss of electrical resistance when the transverse ligament of the upper arm was breached was also recorded. (III) The anesthetic effect was evaluated by other anesthesiologists, and the anesthetic level and effect were measured within 30 minutes after injection. The standard was as follows: excellent: completely painless; good: reduced sensation and mild pain; poor: normal feel and excruciating pain. (IV) The incidence of complications such as perceptual disturbance, vascular puncture injury, hematoma, puncture site pain, pneumothorax, and local anesthesia intoxication during the puncture process was recorded.

### 3.6. Statistical Methods

SPSS 16.0 was employed for analysis and statistics. Normally distributed measurement data were expressed as mean plus or minus standard deviation, and single-factor analysis of variance was used for comparison between groups. Nonnormally distributed measurement data were expressed as median and interquartile range, rank sum test rate was expressed as percentage (%), and Chi-square test was used. Chi-square test was also used for grade data. *P* < 0.05 suggested that the difference was statistically significant.

## 4. Results

### 4.1. Visual Evaluation of the Accuracy of Deep Learning Model Images and Non-AI Images

The prototype of the scanned object with “tomography” was shown clearly, so that the doctor can identify it. In Figure 3, the scapula reached the cutoff frequency after being filtered by Gaussian low-pass. When the filter dropped to a certain value, the boundary was clearly demarcated, leaving a clear barrier between it and its surroundings.

In Figure 4, the second enhancement made the dark part of the scanned object and the background next to it have better contrast, and the color layering was obvious, which can clearly highlight the characteristics of the main part.

Figure 5 shows a group of images of patients with fractures. In the image before enhancement and optimization, the fracture at the bottom right of Figure 5 does not seem to be obvious. If it was not enhanced, it was easy to be misjudged as a nonfracture site and affect the doctor's judgment, while the enhanced ultrasound image can clearly show the location of the fracture.

The second boundary enhancement focused on the optimization of some edge contours and the increase of contrast, which further brought the segmented image closer to the real value.  Figure 6 shows the enhancement curve of accuracy.

### 4.2. The Relationship between the Location of the Traditional Nerve Block in the Scapula Region and the Actual Surface Location of the Ultrasound Scapula Region

The location of the traditional nerve in the scapula region overlapped with the actual body surface location of the nerve in the scapula region under ultrasound, accounting for 60%. The traditional location of the nerve in the scapula region was 38% outside the actual body surface position of the nerve in the scapula region under ultrasound. The traditional location of the nerve in the scapula region was 2% inside the actual body surface position of the nerve in the scapula region under ultrasound (Figure 7). The traditional positioning of the body surface of the scapula region was 0.63 cm away from the actual body surface of the scapula region under ultrasound. The location area of traditional and artificial intelligence ultrasound overlapped greatly, and the location area of artificial intelligence outside is about 36% more than that of the inside.

### 4.3. Comparisons of Injection Time and the Distance between the Puncture Point and the Scapula between the Two Groups

In the contrast group (artificial intelligence ultrasound positioning), it took an average of 7.7 ± 2.1 min from the time the puncture needle touched the skin to the completion of the injection. The operation time of the control group (anatomical positioning) averaged 10.7 ± 2.4 min, and there was a significant difference between the two groups (*p* < 0.05). The actual puncture depth of the contrast group was 62.5 ± 7.2 mm, and that of control group was 79.8 ± 8.9 mm. The difference between the two groups was significant (*p* < 0.05) (Figure 8).

### 4.4. Comparison of the Effects of the Motion Block between the Two Groups

The score of motion block effect in the contrast group and the control group is shown in Figure 9. The scores of clenched fist, elbow flexion, wrist extension, and arm lift were significantly different between the contrast group and the control group, and the motion block effect of the contrast group was better, with statistical difference (*P* < 0.05).

### 4.5. Comparison of Adverse Events during Puncture between the Two Groups

The number of needle tracks needed to be adjusted during puncture in the control group was 3.25 ± 1.36 times, and that in the contrast group was 2.11 ± 1.31 times. *P*=0.009, with statistical difference. The times of encountering bone during puncture were 1.91 ± 1.34 times and 0.68 ± 0.73 times in the two groups, respectively, *P*=0.002, with a statistical difference (Figure 10).

### 4.6. Evaluation of the Anesthesia Effect of the Two Groups

In the contrast group, there were 11 cases with excellent anesthesia effect and 9 cases with good anesthesia. There were 13 cases with excellent anesthesia effect and 7 cases with good anesthesia in the control group (Figure 11). The results showed that the anesthesia effect score of the contrast group was high and the anesthesia effect was good.

### 4.7. Comparison of Puncture Sites and Puncture Adverse Reactions between the Two Groups of the Regional Nerve Block

In Figures 12 and 13, one patient in the control group had a transient abnormal sensation during puncture, while the contrast group did not show transient abnormal sensation. One case in the contrast group was found to have vascular injury, and hematomas were formed during the puncture of the injured blood vessel in the control group. The main complaint of pain during puncture was obvious in the two groups, and there were six patients in the control group, which accounted for 30%. Patients in the contrast group did not have complain of significant pain, and there was a difference between the two groups (*p* < 0.05). There was no pneumothorax and local anesthetic poisoning in the two groups.

## 5. Discussion

The adoption of ultrasonic technology in regional nerve block has become a research hot issue in recent years. Ultrasound technology has produced revolutionary advances in nerve blocks, including the development of spinal regional nerve block [17]. However, there are few reports of the use of ultrasound for nerve block in thoracic paravertebral area. Nowadays, the application of ultrasound technology in clinical regional nerve block has harvested good results and accumulated experience related to real-time guidance of parathoracic region nerve block [18]. In ultrasound, the sagittal section scan block and the oblique section scan block use two modes. The patient can choose the position of the seated side and the position of the decubitus side, as well as the clinical anesthesia area or sitting position. The selection of ultrasonic detection mainly depends on the depth of puncture target and the body shape of the patient, and the weight of the patient has been shown in many studies to be an important factor affecting the depth of thoracic puncture [19]. An ultrasonic probe with the appropriate frequency must be selected by the scanning site. High-frequency linear detection was used for thoracic lateral spinal region nerve block [20]. Ultrasonic imaging is determined by the physical properties of the frequency and wavelength of the ultrasonic wave that detects radiation. Ultrasonic frequency units are related to resolution. The human ear can sense the frequency of sound waves within 20 Hz–20 kHz, and the medical diagnostic frequency of ultrasonic waves is 1–30 MHz. The higher the frequency of ultrasonic detection, the better the transverse resolution. Ultrasound wavelengths mean the distance between adjacent particles in two vibrating regions, allowing a clearer distinction between nerves and surrounding tissue. The longer the wavelength, the higher the transmittance. The frequency of the linear probe is 6–13 MHz, which is suitable for photographing the tissue structure of the body surface. Most of the detection frequencies are 2–7 MHz, which can be used for deep tissue structure imaging [21]. Therefore, the appropriate probe is selected according to the body type of the patient and the depth of the site to be anesthetized. In this study, the body mass of patients was less than 30 kg/m^2^ and good imaging results were obtained using a high-frequency linear probe. The ultrasonic waves emitted by the probes penetrated the surface and propagated into the interior, reflecting the reactions that arouse when obstacles were encountered. Various obstacles can produce different echoes, which are collected and displayed on the screen to get a real-time view of the various parts of the internal organs. In addition, the color Doppler model was combined, which is particularly sensitive to the flow of fluids. Therefore, the blood vessels can be better observed by color Doppler spectroscopy and the flow and diffusion of local anesthesia injection can be observed, which can enable physicians to better conduct the next operation [22].

On the whole, traditional puncture anesthesia lacks the sense of breakthrough during epidural puncture, so the success rate is low and complications are high. A safe and effective guiding puncture method is urgently needed in clinic. The results showed that the fracture site was not obvious in the image before enhancement and optimization, and it was easy to be misjudged as a nonfracture site, affecting the judgment of doctors. The enhanced sonogram clearly showed the fracture location. The localization area of traditional ultrasound and artificial intelligence ultrasound overlapped greatly, and the area of artificial intelligence localization was 36% more than that of inner ultrasound. The algorithm group had fewer puncture needle channels, fewer adverse reactions, and broken operation time, indicating that the ultrasonic positioning effect of the algorithm was better than that of traditional puncture. After the visualization and real-time properties of artificial intelligence ultrasound were used for two control groups, the feasibility of applying ultrasonic image-guided regional nerve block based on deep learning to scapula fracture anesthesia was demonstrated.

## 6. Conclusion

The deep learning-based ultrasound image-guided imaging during scapular fracture surgery with regional nerve block anesthesia was compared with the use of traditional puncture anesthetics. It was proved that the method proposed in this study was more efficient than the traditional method, regardless of whether the method of puncture accuracy evaluation or evaluation of anesthesia effect was used. This method significantly shortened the time required for puncture and reduced complications compared with traditional puncture. In the future, we need to verify the performance of our constructed model in more cases and more disease types. In addition, based on the statistics of various parameters formed by patients using this method, its clinical diagnosis and prognostic predictive effects need to be further studied.

## Figures and Tables

**Figure 1:** Convolutional neural network data analysis model.

**Figure 2:** Image quality gain model.

**Figure 3:** Comparison of the effect of scapula ultrasound before and after the artificial intelligence enhancement. (a) Unenhanced ultrasound image of the scapula. (b) Enhanced ultrasound image of the scapula.

**Figure 4:** Comparison of the effect of scapula CT before and after artificial intelligence enhancement. (a) Unenhanced CT image of the scapula. (b) Enhanced CT image of the scapula.

**Figure 5:** Comparison of scapula fracture before and after ultrasound artificial intelligence enhancement. (a) Unenhanced ultrasound image of the scapula. (b) Enhanced ultrasound image of the scapula.

**Figure 6:** Accuracy enhancement curve.

**Figure 7:** The proportion of the nerve location on the body surface in the scapula region of the traditional method and that under ultrasound.

**Figure 8:** Comparison of puncture time and actual puncture depth between the two groups (*P* < 0.05). (a) Puncture time was compared between the two groups. (b) The puncture depth of the two groups was compared (^*∗*^a considerable difference between groups).

**Figure 9:** The score of motion block effect between the contrast group and the control group (*P* < 0.05) (^*∗*^a considerable difference between groups).

**Figure 10:** Adjustment of the number of needle tracks and the number of bone encounters between the two groups (*P* < 0.05) (^*∗*^a considerable difference between groups).

**Figure 11:** Comparison of anesthesia effect evaluation between the two groups.

**Figure 12:** The puncture site of the regional nerve block in the algorithm group (a) and the ultrasound anatomical diagram after puncture (b).

**Figure 13:** The puncture site (a) of the regional nerve block and the ultrasound anatomy after puncture (b) in the control group. ^*∗*^The bleeding point.

## Data Availability

The data used to support the findings of this study are available from the corresponding author upon request.
